# Hypothermia Protects the Brain from Transient Global Ischemia/Reperfusion by Attenuating Endoplasmic Reticulum Response-Induced Apoptosis through CHOP

This article has been retracted.

**DOI:** 10.1371/journal.pone.0053431

**Published:** 2013-01-03

**Authors:** Xiaojie Liu, Mingshan Wang, Huailong Chen, Yunliang Guo, Fuguo Ma, Fei Shi, Yanlin Bi, Ying Li

**Affiliations:** Department of Anesthesiology, Qingdao Municipal Hospital, Shandong, China; University of Florida, United States of America

## Abstract

Endoplasmic reticulum (ER) stress has been implicated in the pathology of cerebral ischemia. Apoptotic cell death occurs during prolonged period of stress or when the adaptive response fails. Hypothermia blocked the TNF or Fas-mediated extrinsic apoptosis pathway and the mitochondria pathway of apoptosis, however, whether hypothermia can block endoplasmic reticulum mediated apoptosis is never known. This study aimed to elucidate whether hypothermia attenuates brain cerebral ischemia/reperfusion (I/R) damage by suppressing ER stress-induced apoptosis. A 15 min global cerebral ischemia rat model was used in this study. Terminal deoxynucleotidyl transferase-mediated dUTP nick end labeling (TUNEL) positive cells in hippocampus CA1 were assessed after reperfusion of the brain. The expressions of C/EBP-homolo gous protein (CHOP) and glucose-regulated protein 78 (GRP78) in ischemic hippocampus CA1 were measured at 6, 12, 24 and 48 h after reperfusion. The results showed that hypothermia significantly attenuated brain I/R injury, as shown by reduction in cell apoptosis, CHOP expression, and increase in GRP78 expression. These results suggest that hypothermia could protect brain from I/R injury by suppressing ER stress-induced apoptosis.

## Introduction

Hypothermia has been recognized as an effective method in reducing brain injury caused by a variety of neurological insults and may play an important role in emergency brain resuscitation of patients with ischemic stroke, head trauma and cardiac arrest [1], [2], [3], [4], [5]. The neuroprotective effects of mild hypothermia have been well documented in experimental models [6], [7], [8]. The precise mechanisms by which mild hypothermia protects the brain remain to be further elucidated. It is reported that hypothermia prevents cell death by multiple pathways. Among them, hypothermia attenuate cytochrome C (CytC) release and apoptosis [9] including the tumor necrotic factor (TNF) pathway or Fas-mediated extrinsic apoptosis pathway [10]. Earlier studies have found that hypothermia decreases P53 protein levels in the brain which activates genes of apoptosis and pro-apoptotic proteins including Bak,Bax, and PUMA. The Bcl-2 family is much influenced in the way that the pro-apoptotic proteins are inhibited which should have lead to the formation of pores in the mitochondria’s membrane, allowing the release of the cytochrome C to the cytosol, activating caspases, culminating in neuronal death [11], [12], [13]. Zhao [14] reported that biphasic CytC release occurred after transient global ischemia and mild hypothermia protects against ischemic damage by blocking the second phase (12 h, 24 h) of CytC release, possibly by blocking caspases activity. From the above studies, hypothermia can reduce the mitochondria pathway of apoptosis which also known as intrinsic apoptosis pathway. Both the extrinsic and intrinsic apoptosis pathways ultimately activate caspases and then culminate in neuronal death. However, whether hypothermia can block endoplasmic reticulum mediated apoptosis is never known. Recent studies have illustrated the relationship between theendoplasmic reticulum stress(ER) stress and the mitochondria -mediated apoptosis pathway, especially the relationship between bcl-2 family and ER stress [15]. One of the upstream signals that activate these pathways is referred to ER stress. ER is the site for protein synthesis and folding, and also involved in calcium homeostasis and lipid biosynthesis. Many stimuli such as ischemia and hypoxia might perturb ER function resulting in accumulation of unfolded proteins in the ER lumen. This was also known as unfolded proteins response (UPR). Three ER transmembrane receptors named doublestranded RNA-dependent protein kinase-like ER kinase (PERK); inositol requiring enzyme-1 (IRE1) and activating transcription factor (ATF6) are activated to restore ER functions [16]. Firstly, ER chaperones [78-kDa glucose regulated protein (GRP78)] and ER-associated degradation of unfolded proteins as the initially a protective response of UPR. If the stress is prolonged UPR might activate enhancer binding protein homologous protein (chop), caspase-12 and c-Jun N-terminal kinase protein (JNK) [17]. Studies have showed chop is the downstream of all three ER stress pathways and plays an important role in endoplasmic reticulum stress [18]. Prolonged ER stress is implicated in the pathogenesis of ischemia and CHOP plays an important role in the cerebral ischemic damage induced by neuronal death. Up to now, there are no prior studies examining the effects of hypothermia on the ER stress induced apoptotic pathway after transient global ischemia, so we explored these apoptotic events after transient global ischemia, and investigated the effects of hypothermia hypothermia against transient global ischemia through ER stress pathway in the transient global cerebral ischemia model.

## Materials and Methods

### 2.1 Subjects

The study was approved by Qingdao Municipal Hospital Animal Ethics Committee. All the experimental procedures were conducted in conformity with the guidance suggestions for the care and use laboratory animals formulated by the Ministry of Science and Technology of the People’s Republic of China [19]. A total of 273 male Wistar rats (220 to 260 g) supplied by Qingdao Institute of Drug Control were used. Of these, 129 rats were withdrawn from the study for various reasons: 4 died from anesthesia; 27 died during electrocautery of vertebral arteries; 68 died during global ischemia; 19 died during the post surgical period. And 11 rats were paralyzed in vetebral arteries electrocauterizaed. The other 144 rats were randomly divided into global cerebral ischemia/reperfusion group (n = 48), hypothermia group (n = 48) and sham group (n = 48). Core body temperatures were monitored with a rectal probe throughout the surgical procedure. At 6, 12, 24 and 48hours after reperfusion, 6 rats from each group were sacrificed for histological staining, tunnel staining and immunohistochemistry. The other 6 rats were sacrificed for western blot analysis. GRP78 and CHOP expression were measured by immunohistochemistry and western blot analysis.

### 2.2 Surgeries

Rats were starved for 12 h prior to surgery, and then anesthetized by injecting of 10% chloral hydrate (0.35 ml/100 g) intraperitoneally. A model of transient, bilateral hemispheric ischemia was established according to previously described methods [20]. Briefly, vertebral arteries were electrocauterized to induce permanent occlusion. The common carotid arteries were exposed, isolated, and marked using a cotton thread loop. After 24 hours, the exposed bilateral common carotid arteries of the anesthetized rats rats were blocked by artery clamps .After 15 min of ischemia, the clamps were removed to allow reperfusion. A needle electrode was inserted subcutaneously from the parietal region, and connected with the ED-Swan Mark electroencephalo-gram system (Nihon Kohden, Tokyo, Japan). The criteria of successful model were that rats presented unconscious, bilateral dilation of pupils, loss of spontaneous voluntary movements and the righting reflex throughout the ischemia and initial reperfusion periods. As the rats were anesthetized, we mainly rely on EEG. For rats in the hypothermic group, core temperature was decreased to 32–34°C by spraying 100% alcohol onto the rat’s body, and was brought back to normal with a light and a heating pad. Hypothermia maintained for 3 hours after reperfusion. For rats in the sham group, 4 vessels were exposed but without occlusion.

### 2.3 (HE) Staining, Immunohistochemistry and TUNEL Method

The rats (n = 6 at each time point) were deeply anesthetized and intracardially perfused with 0.9% NaCl, followed by 4% paraformaldehyde (PFA). Brains were removed and brain tissues at the coronal plane from 1 to 4 mm posterior to the optic chiasma were harvested. After being fixed for 2 hours, washed for 4 hours, dehydrated with gradient ethanol, cleared with xylene, the brain tissues were embedded with paraffin and cut into 4 µm thickness for hematoxylin and eosin (HE) staining, immunohistochemical staining and TUNEL assay. Anti-rat GRP78 and anti-rat chop polyclonal primary antibody (IgG) were purchased from Santa Cruz Biotechnology. The paraffinized sections were blocked to endogenous peroxidase activity by incubation in distilled water containing 3% hydrogen peroxide for 10 min. Antigen retrieval was performed, using a 0.01 mol/L citrate buffer (pH 6.0) in high pressure cooker for 10 min. Anti GRP78 and anti chop antibody used at a dilution of 1∶150 and 1∶100, respectively, in 2% BSA/PBS were added on the slides and incubated at 37°C for 1 hour. GRP78 and chop were detected with HRP-Polymer anti-Rabbit IgG for 1 h at room temperature. The peroxidase binding sites were detected by staining with diaminobenzidine (DAB). Finally, staining was performed using hematoxylin for 3 secs and observed by microscopy. TUNEL method was performed as described previously [21]. Briefly; Paraffin sections were de-waxed and hydrated. Followed by 3%H_2_0_2_ at room temperature for 10 minutes. The sections were then digested with fresh diluted proteins K(1∶200) at 37°C for 10 minutes. Then, 1 µl TdT and DIG. d-UTP, together with 18 µl marker buffer, were added to each section at 37°C for 2 hours. The sections were then blocked at room temperature for 30minutes,followed by incubation with biotinylated anti-digoxin antibody(1∶200) at 37°C for 30 minutesSABC(1∶100) at 37°C for 30 minutes, DAB coloration, and observation by microscopy..

### 2.4 Western-blots

Animals were perfused transcardially with normal saline, the brains were quickly removed and the hippocampal CA1region was rapidly dissected. The bilateral hippocampus tissues were separated and homogenized with RIPA Lysis Buffer (Beyotime Biotechnology, China). Protein concentrations were determined with a bicinchoninic acid (BCA) protein assay kit (Beyotime Biotechnology, China). Equal amounts of protein samples (total protein extracts, after centrifugation at 12,000 g at 4°C for 5 min. Then, the protein was mixed with buffer and heated at 99°C for 5 min. For western blot analysis an equal amount of protein (50–100 µg) was loaded in each well and subjected to 10% sodium dodecylsulfate-polyacrylamide gel electrophoresis (SDS-PAGE). Separated proteins were then transferred from the gel to polyvinylidinene fluoride (Millipore, Bedford, MA, USA) membranes and blocked in 5% non-fat dry milk prepared in 1× TBST. The membranes were incubated with the primary antibodies overnight at 4°C. The following primary antibodies were used: GRP78(1∶200, Santa Cruz Biotechnology, Santa Cruz, CA, USA), CHOP (1∶100, Santa Cruz Biotechnology, CA, USA) or GAPDH antibody (1∶1000, Zhongshan Goldenbridge Biotechnology, China). After washing primary antibodies with 1×TBST, the membranes were incubated with appropriate secondary antibodies for 2 h at room temperature. The blots were developed using ECL (Beyotime Institute of Biotechnology, China).

### 2.5 Statistics

All data were expressed as mean ± standard deviation (SD) and analyzed by SPSS 13.0. Repeated measures ANOVA was used as appropriate for comparison between different groups followed by post hoc test for multiple comparisons. *P<0.05* was considered as statistically significant.

## Results

### 3.1 Hippocampus Neuronal Morphology

Compared with sham group, the number of normal neurons in hippocampus CA1 area decreased in ischemia and hypothermia group. And the number of neurons with nuclear pyknosis increased significantly in hippocampus CA1 area from ischemia and hypothermia group. What’s more, compared with hypothermia group, the neuronal degeneration in ischemia group is more severe at each time points from ischemia group. At reperfusion 48 hours, the number of survival neurons in hypothermia group is more than in ischemia group (Fig. 1).

**Figure 1:** Neurons in hippocampus CA1 area. (a) The picture showed the neurons in hippocampus CA1 area. The neurons in sham group (A) displayed regular appearance with large and round nuclei but pyknosis was observed in ischemia (C) and hypothermia group (B). (b) Compared with sham group(89.3±6.1) (A), the number of normal neuronal is fewer and the neurons of morphologic abnormality is more in ischemia group(47.3±4.5) (C). The number of survival neurons in hypothermia group(64.5±7.5) (B) is more than that in ischemia group. /400×visual field.

The neurons in sham group (A) displayed regular appearance with large and round nuclei but pyknosis was observed in ischemia(C) and hypothermia group (B).

Compared with sham group (89.3±6.1) (A), the number of normal neuronal is fewer and the neurons of morphologic abnormality is more in ischemia group (47.3±4.5) (C). The number of survival neurons in hypothermia group (64.5±7.5) (B) is more than that in ischemia group. /400×visual field.

### 3.2 The Expression of GRP78 and Chop

The expression of chop and GRP78 protein neurons was found in hippocampus CA1 after cerebral ischemia reperfusion (Fig. 2, 3). In normothermic and mild hypothermic ischemia groups, the optical densities of chop and GRP78 in hippocampus CA1 neurons at 6, 12, 24 and 48hour reperfusion following 15 minute ischemia (15 min/6 h, 15 min/12 h, 15 min/24 h, 15 min/48 h respectively) were showed in Fig. 2, 3. Mild hypothermia decreased the expression of GRP78 protein and increased the expression of chop protein. Immunohistochemistry showed the GRP78 was barely detected in sham group (A). The expression of GRP78 in hypothermia group (B) is much stronger than that in ischemia group (C) at reperfusion 24 hours. /400×visual field.

**Figure 2:** Expression of GRP78 in hippocampus CA1. (a) Immunohistochemistry showed the GRP78 was barely detected in sham group (A). The expression of GRP78 in hypothermia group (B) is much stronger than that in ischemia group (C) at reperfusion 24 hours. /400×visual field (b) Western blot analysis showed that the GRP78 was barely detected in sham group. In brains of ischemia group, it was increased 6 hour after 15 min of ischemia and gradually decreased thereafter; however, the degree of increase was much bigger in the hypothermia brains. (c) Quantitative analysis of Western blotting showed that hypothermia after ischemia significantly increased GRP78 after 15 minutes of ischemia (*P<0.05* compared with ischemia brains at the same time points, 6 rats from each group at every time points were used for analysis).

**Figure 3:** Expression of chop in hippocampus CA1. (a) Immunohistochemistry showed the chop was barely detected in sham group (A).The expression of chop in hypothermia group (B) is much weaker than that in ischemia group (C) at reperfusion 24 hours. /400×visual field (b) Western blot analysis showed that the chop was barely detected in sham group. In brains of ischemia group, it was increased 6 hour after 15 minutes of ischemia and gradually decreased thereafter; however, the degree of increase was much smaller in the hypothermia brains. (c) Quantitative analysis of Western blotting showed that hypothermia after ischemia significantly decreased chop after 15 minutes of ischemia (P<0.05 compared with ischemia brains at the same time points. 6 rats from each group at every time points were used for analysis).

Western blot analysis showed that the GRP78 was barely detected in sham group. In brains of ischemia group, it was increased 6 hour after 15 min of ischemia and gradually decreased thereafter; however, the degree of increase was much bigger in the hypothermia brains.

Quantitative analysis of Western blotting showed that hypothermia after ischemia significantly increased GRP78 after 15 minutes of ischemia (*P<0.05* compared with ischemia brains at the same time points, 6 rats from each group at every time points were used for analysis). Immunohistochemistry showed the chop was barely detected in sham group (A). The expression of chop in hypothermia group (B) is much weaker than that in ischemia group (C) at reperfusion 24 hours. /400×visual field.

Western blot analysis showed that the chop was barely detected in sham group. In brains of ischemia group, it was increased 6 hour after 15 minutes of ischemia and gradually decreased thereafter; however, the degree of increase was much smaller in the hypothermia brains.

Quantitative analysis of Western blotting showed that hypothermia after ischemia significantly decreased chop after 15 minutes of ischemia (P<0.05 compared with ischemia brains at the same time points. 6 rats from each group at every time points were used for analysis).

### 3.3 TUNEL

TUNEL positive staining was absent in the sham groups (Fig. 4), and there were few TUNEL positive cells among the hypothermia group (Fig. 4). However, many positive cells could be observed in the ischemia group (Fig. 4). Detection of apoptosis in hippocampus CA1 pyramidal neurons was carried out using TUNEL staing. The sham group showed a large number of neurons and almost no TUNEL-positive cells (5.1±1.2) (A). In ischemia (C) and hypothermia (B) groups, the number of neurons was decreased and substantial TUNEL-positive cells were detected. The number of TUNEL-positive cells in hypothermia group (34.4±4.2) (B) is more than in ischemia group (40.5±5.7) (C), /400×visual field.

**Figure 4:** Neuronal apoptosis in CA1 region of hippocampus induced by global cerebral ischemia. Detection of apoptosis in hippocampus CA1 pyramidal neurons was carried out using Tunel staing. The sham group showed a large number of neurons and almost no TUNEL-positive cells (5.1±1.2) (A). In ischemia (C) and hypothermia (B) groups, the number of neurons were decreased and substantial TUNEL-positive cells were detected. The number of TUNEL-positive cells in hypothermia group (34.4±4.2) (B) is more than in ischemia group (40.5±5.7) (C), /400×visual field.

## Discussion

It has been reported that hypothermia blocked the TNF pathway of apoptosis or extrinsic Fas-mediated apoptosis pathway and the mitochondria pathway of apoptosis. However, whether hypothermia can block endoplasmic reticulum mediated apoptosis is never known. This study confirms that mild hypothermia for 3 h after global ischemia protects hippocampus neurons from a global ischemic insult, and demonstrates that this protection following global ischemia is associated with reduced apoptosis as assessed by TUNEL staining. Furthermore, we showed for the first time that mild hypothermia was associated with increased GRP78 expression and decreased chop expression suggesting a mechanism for the observed neuroprotection.

ER is the site for protein synthesis and folding, and also involved in calcium homeostasis and lipid biosynthesis. Cerebral ischemia causes severe ER stress that results in ER function disruption and unfolded proteins accumulation in the ER lumen called unfolded protein reaction UPR [22], ultimately leads to cell death [23]. Apoptosis initiated by ER stress is largely dependent on the release of cytochrome c from the mitochondrial intermembrane space into the cytosol.

Brain I/R injury up-regulates the expression of ER stress markers such as CHOP and GRP78 [24] that results in ER stress-associated apoptosis [25]. Similar to their studies, our results also demonstrated that I/R injury increases CHOP expression, GRP78 induction and apoptosis in the hippocampus after cerebral ischemia. The ER chaperone GRP78 (glucose-regulated protein of 78 kDa) with antiapoptotic properties is a central regulator of ER homeostasis, and its up-regulation is widely used as a sentinel marker for ER stress under pathologic conditions. As a major ER chaperone, GRP78 facilitates protein folding, preventing intermediates from aggregating and promoting misfolded protein for proteasome degradation [20]. Our result has revealed the activation of GRP78 started at 6 h after ischemia and reached the peak at 24 h after ischemia attack. Compared with the ischemia group, the amount of GRP78 expression in hypothermia group is much more than that in ischemia group which is in. consistent with the finding of Masayuki Aoki [26], [27]. There was a significant reduction in the number of TUNEL-positive cells in the hippocampus CA1 in the hypothermia group rats at 48 h of reperfusion in our study. Therefore, we believe that the increased GRP78 expression contributes to the hypothermia-induced neuroprotection in hippocampus area against cerebral ischemia. It has been reported that CHOP^−/−^mice exhibit reduced apoptosis in response to ER stress and have smaller infarcts than wild-type animals subjected to bilateral carotid artery occlusion [28], [29]. Thus, CHOP is the downstream of ER stress induced apoptosis [30], [31]. Further, our results showed that mild hypothermia significantly decreased the activation of CHOP at 24 h of reperfusion. In agreement with the study of Wang, our study showed the increased expression of GRP78 attenuated the induction of CHOP during ER stress and reduced ER stress-induced apoptosis when hypothermia was applied after global ischemia [32]. Previous studies have suggested that CHOP sensitizes cells to ER stress induced-apoptosis through down-regulation of the anti-apoptotic factor B cell lymphoma-2 (Bcl-2) and up-regulation of reactive oxygen species (ROS) [14], [23]. However, numerous studies have certificated the neuroprotection of hypothermia by reducing the oxidative stress, lipid peroxidation, glutamate excitotoxicity together with increased the anti-apoptotic protein Bcl-2 [33]. We hypothesize that some molecules of CHOP pathway, such as Bcl-2 and ROS, may contribute to the decreased TUNEL-positive cells by hypothermia. We already have known that the permeabilization of the mitochondrial outer membrane (MOM) and the consequent release of cytochrome c are regulated by a group of proteins known as the Bcl-2protein families. Collectively, the Bcl-2 protein family monitors incoming stress signals and orchestrates the initiation of the mitochondrial or intrinsic pathway to apoptosis. Bcl-2 has previously shown that it’s suppress cell death by inhibiting free radical production and prevent the release of cytochrome C from mitochondria and block caspase activation [34], [35], [36]. But the intrinsic relationship among them induced by hypothermia following global ischemia needs to be further studied.
